The article "Mannitol increases renal blood flow and maintains filtration fraction and oxygenation in postoperative acute kidney injury: a prospective interventional study" was published in 2012. Journal: Crit Care.

# Mannitol increases renal blood flow and maintains filtration fraction and oxygenation in postoperative acute kidney injury: a prospective interventional study

**DOI:** 10.1186/cc11480

**Published:** 2012-08-17

**Authors:** Gudrun Bragadottir, Bengt Redfors, Sven-Erik Ricksten

**Affiliations:** 1 Department of Anaesthesiology and Intensive Care Medicine, Sahlgrenska Academy, University of Gothenburg, Sahlgrenska University Hospital, SE-413 45 Gothenburg, Sweden

## Abstract

**Introduction:**

Acute kidney injury (AKI), which is a major complication after cardiovascular surgery, is associated with significant morbidity and mortality. Diuretic agents are frequently used to improve urine output and to facilitate fluid management in these patients. Mannitol, an osmotic diuretic, is used in the perioperative setting in the belief that it exerts reno-protective properties. In a recent study on uncomplicated postcardiac-surgery patients with normal renal function, mannitol increased glomerular filtration rate (GFR), possibly by a deswelling effect on tubular cells. Furthermore, experimental studies have previously shown that renal ischemia causes an endothelial cell injury and dysfunction followed by endothelial cell edema. We studied the effects of mannitol on renal blood flow (RBF), glomerular filtration rate (GFR), renal oxygen consumption (RVO_2_), and extraction (RO_2_Ex) in early, ischemic AKI after cardiac surgery.

**Methods:**

Eleven patients with AKI were studied during propofol sedation and mechanical ventilation 2 to 6 days after complicated cardiac surgery. All patients had severe heart failure treated with one (100%) or two (73%) inotropic agents and intraaortic balloon pump (36%). Systemic hemodynamics were measured with a pulmonary artery catheter. RBF and renal filtration fraction (FF) were measured by the renal vein thermo-dilution technique and by renal extraction of chromium-51-ethylenediaminetetraacetic acid (^51^Cr-EDTA), respectively. GFR was calculated as the product of FF and renal plasma flow RBF × (1-hematocrit). RVO_2 _and RO_2_Ex were calculated from arterial and renal vein blood samples according to standard formulae. After control measurements, a bolus dose of mannitol, 225 mg/kg, was given, followed by an infusion at a rate of 75 mg/kg/h for two 30-minute periods.

**Results:**

Mannitol did not affect cardiac index or cardiac filling pressures. Mannitol increased urine flow by 61% (*P *< 0.001). This was accompanied by a 12% increase in RBF (*P *< 0.05) and a 13% decrease in renal vascular resistance (*P *< 0.05). Mannitol increased the RBF/cardiac output (CO) relation (*P *= 0.040). Mannitol caused no significant changes in RO_2_Ext or renal FF.

**Conclusions:**

Mannitol treatment of postoperative AKI induces a renal vasodilation and redistributes systemic blood flow to the kidneys. Mannitol does not affect filtration fraction or renal oxygenation, suggestive of balanced increases in perfusion/filtration and oxygen demand/supply.

## Introduction

Acute kidney injury (AKI) complicates 15% to 30% of cardiac surgeries and is associated with significant morbidity and mortality [1-4]. Even minor changes in serum creatinine are associated with increased inpatient mortality [5,6]. Impaired renal oxygen delivery, caused by intraoperative hypotension and hemodilution-induced anemia and postoperative low cardiac output, is considered to be the cause of postoperative AKI in this group of patients [4,7]. The renal medulla is at the border of hypoxia under normal conditions, due to the concentration mechanism, and therefore particularly sensitive to ischemia [8,9].

It was recently shown that renal oxygenation (renal oxygen supply/demand relation) is severely impaired in patients with early AKI after complicated cardiac surgery [10], in turn, caused by a 50% increase in renal vascular resistance, compared with uncomplicated postcardiac-surgery patients. From experimental studies, it has been suggested that renal vasoconstriction in AKI is caused by afferent arteriolar vasoconstriction mediated by the tubuloglomerular feedback mechanism, vasoconstrictors (catecholamines, angiotensin II, endothelin), and outer medullary congestion. Furthermore, it has been ascribed to ischemic endothelial cell injury, causing an imbalance in the production of endothelin and endothelial nitric oxide, or to angiotensin II-induced activation of reactive oxygen species that inactivates NO [11-13]. Finally, it has been suggested that outer medullary hypoxia may cause endothelial ischemic injury and cell swelling, contributing to congestion and impaired perfusion of this region [14]. It would therefore be logical that interventions that alleviate this afferent arteriolar vasoconstriction would be beneficial, as they could potentially increase RBF and GFR.

Oliguria is a poor prognostic indicator in patients with AKI [15,16], and diuretic agents are frequently used to improve urine output and to facilitate fluid management in these patients. Mannitol, an osmotic diuretic, has been used in the belief that it exerts renoprotective properties in patients undergoing surgery. However, results from studies in which mannitol has been evaluated in the perioperative setting, for prevention or treatment of AKI, are divergent. Although mannitol has failed to show a prophylactic effect in patients undergoing abdominal aortic or cardiac surgery [17,18], mannitol has been shown to reduce the incidence of postoperative AKI in the setting of renal transplantation, along with volume expansion [19,20]. Furthermore, mannitol treatment has been shown to increase the glomerular filtration rate (GFR) in patients after severe trauma or surgery [21]. In addition, our group recently showed that mannitol increases GFR in postoperative cardiac surgery patients [22], possibly by a deswelling effect on tubular cells.

To evaluate in more detail the potential beneficial effects of mannitol for treatment of AKI in the perioperative setting, our aim was to evaluate the effects of mannitol on GFR, renal blood flow (RBF), renal oxygen consumption (RVO_2_), and the renal oxygen supply/demand relation in patients with early, ischemic AKI after complicated cardiac surgery. To this end, we used the retrograde renal vein thermodilution technique and renal extraction of ^51^chromium-ethylene-diaminetetraacetic acid (^51^Cr-EDTA) for rapid bedside estimation of RBF and GFR without the need for urine collection [23]. In the present study, we tested the null hypothesis that mannitol, in clinically used doses, affects neither RBF nor GFR in patients with AKI after cardiac surgery.

## Materials and methods

### Study population

The study protocol was approved by the Human Ethics Committee of the University of Gothenburg. Informed consent was obtained from the patient's next of kin before enrolment in the study. Between September 2007 and October 2011, 13 patients who developed AKI after complicated heart surgery were included in the study according to these inclusion criteria: (a) cardiac surgery with cardiopulmonary bypass; (b) normal preoperative renal function (serum creatinine ≤105 µ*M*); and (c) development of AKI, stage 1 or 2, according to the Acute Kidney Injury Network criteria, defined as a 50% to 200% postoperative increase in serum creatinine from baseline [5]. The following exclusion criteria were used: (a) heart transplantation, thoracoabdominal aortic surgery, (c) aortic dissection, (d) use of nephrotoxic drugs such as radiocontrast agents, aminoglycoside antibiotics, or nonsteroidal antiinflammatory drug (NSAID) analgesics.

In the intensive care unit (ICU), the patients were sedated with propofol (50.1 ± 3.3 μg/kg/min), treated with morphine or fentanyl, and mechanically ventilated to normocapnia. The hemodynamic and renal management of the patients was at the discretion of the attending intensive care physician. The treatment protocol included inotropic support with milrinone and/or norepinephrine to maintain cardiac index ≥2.1 L/min/m^2^, whole-body oxygen extraction ≤40%, and mean arterial pressure (MAP) at 70 to 80 mm Hg, with or without an intraaortic balloon pump. A continuous infusion of furosemide (5 to 40 mg/h) was used, if needed, to promote diuresis. Because all patients were sedated, neurologic status was not included in the sequential organ-failure assessment score (SOFA score) [24].

### Systemic hemodynamics

Arterial blood pressure was measured with a radial or femoral arterial catheter. Systemic hemodynamics were measured with a pulmonary artery thermodilution catheter (Baxter Healthcare Corporation, Irvine, CA, USA). Measurements of thermodilution cardiac output were performed in triplicate and indexed to body surface area to derive the cardiac index (CI). The mean coefficient of variation for measurement of CI was 1.6%. The pulmonary artery wedge pressure (PCWP) was measured intermittently. Systemic vascular resistance index (SVRI), pulmonary vascular resistance index (PVRI), and left ventricular stroke volume index (SVI) were calculated according to standard formulae. Sodium was measured potentiometrically with a sodium electrode (ABL800 Flex; Radiometer, Bronshoj, Denmark). The sensitivity limits of the sodium electrode are 90% to 105%.

### Measurement of renal variables

An 8-Fr catheter (Webster Laboratories, Baldwin Park, CA, USA) was introduced into the left renal vein via the right femoral vein, under fluoroscopic guidance. The catheter was placed in the central portion of the renal vein, and its position was verified with venography, by using ultra-low doses of iohexol, 5 to 15 mg I/kg (Omnipaque 300 mg I/ml; GE Healthcare, Stockholm, Sweden) [25]. The technique for measurement of RBF with retrograde thermodilution has previously been described in detail [22,23,26,27]. The total RBF was assumed to be twice the blood flow to the left kidney. After blood and urine blanks were taken, an intravenous priming dose of ^51^Cr-EDTA (0. 6 MBq/m^2 ^body surface area) was given, followed by an infusion at a constant rate, individualized to body weight and serum creatinine. Serum ^51^Cr-EDTA activities from arterial and renal vein blood were measured with a well counter (Wizard 300, 1480 Automatic Gamma Counter; Perkin Elmer LAS, Turku, Finland). Urine was collected in 30-minute periods to measure urine flow and sodium excretion. An indwelling Foley catheter drained the urine from the bladder. The levels of ^51^Cr-EDTA were obtained from arterial and renal vein blood at the end of each urine-collection period.

### Experimental procedure

The patients were included in the study from 2 to 6 days after the cardiac surgery. After an equilibration period of at least 60 minutes, two 30-minute urine-collection control periods were started, followed by the administration of mannitol, 150 mg/ml (Mannitol; Baxter Viaflo, Baxter Medical AB, Kista, Sweden). The patients received a bolus dose of mannitol, 225 mg/kg, followed by a continuous infusion of mannitol at a rate of 75 mg/kg/h for two 30-minute urine collection periods. Thermodilution measurements of RBF, hemodynamic variables, as well as blood and urine samples, were obtained at the end of each urine-collection period. During the experimental procedure, the blood pressure was kept constant, and an isotonic crystalloid solution was continuously infused to substitute for fluid losses due to the diuretic response.

### Data calculation

RBF was measured with retrograde thermodilution of the left renal vein. FF was measured with renal extraction of ^51^Cr-EDTA, (arterial-renal vein)/arterial ^51^Cr-EDTA concentration). A significant error in the calculation of renal extraction of filtration markers, by using this formula, may occur in situations with high diuresis and a relatively low renal plasma flow [28]. Renal ^51^Cr-EDTA extraction and RBF values were therefore corrected by taking the urine flow into account [28]. GFR was calculated as the product of FF and renal plasma flow (FF × RBF × (1-hematocrit). Renal vascular resistance (RVR) was calculated from the formula RVR = (MAP-CVP)/RBF. RVO_2 _and renal oxygen extraction (RO_2_Ex) were derived from the formulas RVO_2 _= RBF × (CaO_2_-CvO_2_) and RO_2_Ex = (CaO_2_-CvO_2_/CaO_2_), respectively, where CaO_2 _and CvO_2 _are the arterial and renal vein oxygen contents. All renal data were normalized to a body surface area of 1.73 m^2^. The glomerular filtration of sodium (GF_Na_) was calculated from the formula GF_Na _= GFR × P_Na_, and the tubular reabsorption of sodium (TR_Na_) was defined as the difference between the filtered load of sodium and the renal sodium excretion (that is, TR_Na _= GF_Na _- (U_Na _× U_V_)). Fractional excretion of sodium (FE_Na_) was defined as (U_Na _× U_V_)/GF_Na_

### Statistical analysis

Based on our previous study [22], we calculated that 10 patients had to be included to detect a mannitol-induced change in GFR of 20%, at a power of 80% and at a significance level of 0.05, with a standard deviation of 12.2 ml (paired design). Data on renal and hemodynamic variables from the two control periods (C1, C2), as well as the two mannitol-treatment periods (M1, M2) were pooled. The renal and hemodynamic effects of mannitol, compared with control, were assessed with a paired *t *test. A probability level (*P *value) of less than 0.05 was considered to indicate statistical significance. The data are presented as mean ± standard error of the mean (mean ± SEM).

## Results

Thirteen patients were included in the study. Two patients were excluded from the study because of unsuccessful placement of the renal vein catheter. In total, 11 patients were thus evaluated. Baseline characteristics of the patients are presented in Table 1. Serum creatinine had increased by 52% to 158% at the day of study. The patients had a mean SOFA score of 9 (range, 7 to 12). All patients were treated with norepinephrine infusion. Eight (73%) patients were treated with milrinone, 10 (91%) patients had furosemide infusion, and four (36%) patients needed an IABP (Table 2). Two (18%) patients required continuous renal-replacement therapy, and five (45%) patients died during their ICU stay.

**Table 1:** Baseline characteristics

Preoperative characteristics	
Gender, *n *(% men)	8 (73)
Age (years)	67.1 ± 1.80
BSA (m^2^)	2.1 ± 0.09
Preop LVEF (%)	41.4 ± 5.56
Diabetes, type 2 (%)	2 (18)
Hypertension, *n *(%)	7 (64)
Serum creatinine (µ*M*)	86.3 ± 3.41

Preoperative treatment	

ACE inhibitor, *n *(%)	8 (73)
β-Adrenergic blocker, *n *(%)	10 (90)
Calcium antagonists, *n *(%)	1 (9)
Euroscore	7.4 ± 1.39

Perioperative characteristics	

Type of surgery	
CABG, *n *(%)	3 (27)
Valve, *n *(%)	4 (36)
Combined, *n *(%)	3 (27)
Other, *n *(%)	1 (9)
Nonelective, *n *(%)	4 (36)
CPB time (minutes)	138.1 ± 13.9
Aortic cross-clamp time (minutes)	80.8 ± 11.0
ICU Higgins risk score	9.0 ± 1.46

Data are presented as mean ± SEM. ACE, angiotensin-converting enzyme; BSA, body surface area; CABG, coronary artery bypass surgery; CPB, cardiopulmonary bypass; ICU, intensive care unit; LVEF, left ventricular ejection fraction; nonelective, surgery performed within 24 hours after referral; Preop, preoperative.

**Table 2:** Individual data at inclusion to the study

Patient number	Study entry (day)	Preop. creatinine (µ*M*)	Inclusion creatinine (µ*M*)	Creatinine increase (%)	SOFA score	IABP	Norepinephrine (µg/kg/min)	Milrinone (µg/kg/min)	Furosemide (µg/kg/min)
1	4	91	151	66	12	No	0.14	0.18	0
2	4	102	170	67	7	No	0.09	0	0.99
3	2	90	146	62	10	Yes	0.33	0.44	3.70
4	6	93	210	126	7	No	0.32	0.25	1.05
5	5	84	217	158	9	No	0.27	0	0.95
6	2	82	135	65	10	No	0.33	0.26	3.21
7	2	102	155	52	10	Yes	0.92	0.26	7.41
8	4	83	182	119	10	No	0.95	0.20	6.53
9	2	81	127	57	6	Yes	0.39	0.40	2.22
10	4	62	150	141	10	Yes	0.21	0.50	1.14
11	5	79	163	107	8	No	0.40	0	5.55

Mean	3.83	90.3	164	93	9.0	36%	0.39	0.31*	1.98*
SEM	0.43	3.41	8.67	11.55	0.54		0.09	0.04*	0.78*

IABP, intraaortic balloon pump; Preop, preoperative; SOFA, sequential organ-failure assessment. *Mean and SEM among treated.

Data obtained during the two control periods, C1 and C2, did not differ in any of the measured variables.

### Effects of mannitol on systemic hemodynamic variables

Mannitol induced a significant increase in SVI (4%) and significantly decreased Hct (2%) (Table 3). Mannitol caused no significant changes in MAP, MPAP, CI, HR, SVRI, or PVRI and had no effects on filling pressures (CVP, PCWP). The body temperature did not change during the experimental procedure.

**Table 3:** Effects of mannitol on systemic hemodynamic variables

	C1	C2	M1	M2	*P *value
MAP (mm Hg)	76.0 ± 1.30	75.4 ± 1.43	75.3 ± 0.91	74.6 ± 1.29	0.467
CI (L/min/m^2^)	2.9 ± 0.20	2.9 ± 0.21	3.0 ± 0.21	3.0 ± 0.21	0.109
SVI (ml/beat/m^2^)	30.5 ± 2.57	31.1 ± 2.63	31.8 ± 2.68	32.2 ± 2.55	0.046
HR (beats/min)	99.5 ± 5.78	97.1 ± 4.87	96.7 ± 4.99	96.0 ± 4.77	0.190
SVRI (dynes s/cm^5^/m^2^)	1,794 ± 112	1,776 ± 138	1,738 ± 124	1,708 ± 132	0.074
PVRI (dynes s/cm^5^/m^2^)	272 ± 26.6	278 ± 26.0	269 ± 22.9	260 ± 17.0	0.573
CVP (mm Hg)	12.6 ± 1.02	13.2 ± 0.90	13.2 ± 1.07	13.0 ± 1.04	0.531
MPAP (mm Hg)	27.1 ± 2.21	27.2 ± 2.00	27.3 ± 2.16	26.9 ± 2.06	0.933
PCWP (mm Hg)	17.3 ± 2.00	17.3 ± 1.95	17.5 ± 2.09	17.4 ± 2.02	0.720
Hct	0.313 ± 0.015	0.316 ± 0.012	0.309 ± 0.012	0.309 ± 0.013	0.012
Body temperature (^o^C)	37.55 ± 0.23	37.58 ± 0.21	37.54 ± 0.20	37.50 ± 0.19	0.182

Data are presented as mean ± SEM. C1, first control period before mannitol infusion; C2, second control period before mannitol infusion; CI, cardiac index; CVP, central venous pressure; Hct, hematocrit; HR, heart rate; M1, first period with mannitol infusion (150 mg/ml, infusion rate of 0.5 ml/kg/h); M2, second period with mannitol infusion (150 mg/ml; infusion rate of 0.5 ml/kg/h); MAP, mean arterial pressure; MPAP, mean pulmonary artery pressure; PCWP, pulmonary capillary wedge pressure; PVRI, pulmonary vascular resistance index; SVI, stroke volume index; SVRI, systemic vascular resistance index.

### Effects of mannitol on renal variables

Mannitol induced a significant increase in RBF (12%) and significantly decreased RVR (-13%) (Table 4 and Figure 1). Mannitol increased the RBF/CO relation (*P *= 0.040). Mannitol also caused significant increases in urine output (61%) and FE_Na _(58%). Although mannitol tended to increase GFR (16%, *P *= 0.16), sodium filtration (18%, *P *= 0.14), tubular sodium reabsorption (14%, *P *= 0.28), and RVO_2 _(10%, *P *= 0.14), none of these changes reached statistical significance. Mannitol affected neither FF nor RO_2_Ext.

**Table 4:** Effects of mannitol on renal variables

	C1	C2	M1	M2	*P *value
RBF (ml/min)	472 ± 48	465 ± 44	521 ± 49	503 ± 47	0.016
RVR (mm Hg/ml/min)	0.150 ± 0.018	0.147 ± 0.015	0.132 ± 0.014	0.135 ± 0.014	0.030
GFR (ml/min)	33.8 ± 4.6	36.0 ± 5.56	41.0 ± 7.28	39.2 ± 5.69	0.156
FF	0.104 ± 0.015	0.113 ± 0.016	0.110 ± 0.016	0.103 ± 0.011	0.743
GFNa (mmol/min)	4.82 ± 0.66	5.05 ± 0.82	5.98 ± 1.08	5.61 ± 0.82	0.141
TRNa (mmol/min)	4.45 ± 0.64	4.65 ± 0.79	5.30 ± 1.04	5.00 ± 0.79	0.286
FENa	0.078 ± 0.023	0.089 ± 0.023	0.125 ± 0.025	0.117 ± 0.021	0.008
RVO_2 _(ml/min)	10.62 ± 1.25	11.35 ± 1.27	12.1 ± 1.48	11.5 ± 1.30	0.138
RO_2_Ex	0.169 ± 0.014	0.174 ± 0.014	0.172 ± 0.016	0.170 ± 0.017	0.940
Urine flow (ml/min)	3.50 ± 0.68	3.58 ± 0.58	6.01 ± 1.09	5.38 ± 0.99	0.004
RBF/CO	0.080 ± 0.009	0.080 ± 0.008	0.088 ± 0.009	0.084 ± 0.008	0.040

Data are presented as mean ± SEM. C1, first control period before mannitol infusion; C2, second control period before mannitol infusion; FENa, fractional excretion of sodium; FF, filtration fraction; GFNa, sodium filtration; GFR, glomerular filtration rate; M1, first period with mannitol infusion (150 mg/ml, infusion rate of 0.5 ml/kg/h); M2, second period with mannitol infusion (150 mg/ml, infusion rate of 0.5 ml/kg/h); RBF, renal blood flow; RO_2_Ex, renal oxygen extraction; RVR, renal vascular resistance; RVO_2_, renal oxygen consumption; TRNa, sodium reabsorption.

**Figure 1:** **Effects of mannitol (M1, M2) on renal vascular resistance (RVR), renal blood flow (RBF), glomerular filtration rate (GFR), and renal filtration fraction (FF)**. *P < 0.05.

## Discussion

The main findings of the present study on cardiac surgery patients with postoperative early AKI were that mannitol induced a renal vasodilatation and increased RBF with no changes in filtration fraction or the renal oxygen supply/demand relation, as assessed by the lack of effect on RO_2_Ex.

To our knowledge, no previous studies exist on the effects of mannitol on renal perfusion, filtration, and oxygenation in patients with AKI. In most animal studies, it has been shown that mannitol increases RBF by renal vasodilation during both normotensive [29-31] and hypotensive conditions [32-34]. Data on the effects of mannitol on RBF in humans, however, are scarce. With the xenon^133 ^washout technique, Castaneda-Zuniga *et al*. [35] studied the effects of mannitol (20%) infusion on RBF in humans and demonstrated only a minimal increase in RBF. With the same methods as in the present study, Kurnik *et al*. [36] studied the effect of mannitol (15%) on RBF in patients with moderate chronic renal failure and found that mannitol did not affect RBF. Those results are supported by a study, recently published by our group, demonstrating no effect of mannitol on RBF, in postoperative uncomplicated cardiac surgery patients with normal renal function [22].

What are the mechanisms behind the mannitol-induced decrease in RVR in early clinical, ischemic AKI, as demonstrated in the present study? It has been suggested that the mannitol-induced renal vasodilatory response to experimental renal ischemia is mediated directly by increased synthesis of prostacyclin, or indirectly by augmenting plasma levels of ANP because of the plasma volume expansion [34,37]. In the present study, plasma volume expansion with mannitol was not large enough to cause increased cardiac filling pressures at the time of RBF measurements. However, we cannot rule out the possibility that mannitol bolus plus infusion induced a transient increase in cardiac filling pressures and distention, causing a release of natriuretic peptides. In our previous study in postoperative uncomplicated cardiac patients with normal renal function, by using an identical protocol, we found that mannitol did not affect RBF [22], suggesting that mannitol-induced plasma volume expansion and the consequent cardiac release of renal vasodilatory cardiac peptides is not the main mechanism behind the renal vasodilation, as demonstrated in the present study.

Experimental studies have shown that renal ischemia causes endothelial cell injury and dysfunction followed by endothelial cell edema [14]. Flores *et al*. [38] showed in an animal study that ischemia-induced endothelial cell swelling can be reversed and prevented by mannitol. They suggested that the failure of blood flow to return to the kidney after transient ischemia, the so-called "no reflow" phenomenon, was due to swollen endothelial cells, and that the no-reflow could be corrected by mannitol. Based on those experimental studies, one could therefore speculate that mannitol might exert its beneficial effect on renal perfusion in patients with AKI by a deswelling effect on injured endothelial cells.

Data on the effects of mannitol on the GFR are divergent. In animal studies, mannitol has been shown to decrease [39], increase [40], or to have no effect on the GFR [29]. In hypoperfused animal kidneys, mannitol infusion tends to restore the GFR toward normal levels [32,33,41], when given both before and after the induction of hypotension [33,41]. Flores *et al*. [38] suggested that mannitol maintains the GFR in renal ischemia primarily by an osmotic effect that reduces vascular endothelial cell swelling, which would reduce RVR and increase RBF. A study on healthy human volunteers showed no effect of mannitol on GFR [42], whereas mannitol increased creatinine clearance in patients with severe trauma/surgery, as shown in a study by Valdes *et al*. [21]. In a recent study on uncomplicated postcardiac-surgery patients with normal renal function, by using a protocol identical to that in the present study, we showed that mannitol induced a 20% increase in GFR and filtration fraction with no change in RBF [22]. Those findings were interpreted as deswelling effect on tubular cells, subjected to intraoperative hypotensive episodes, and recruitment of functional nephrons that are opened up by mannitol, which will increase tubular flow and restore GFR [43]. In the present study, mannitol tended to increase GFR (16%), but the increase in GFR did not reach statistical significance (*P *= 0.16). This study was powered to detect a 20% increase in GFR, based on our previous study [22]. In a *post hoc *power analysis, we found that the sample size would have to be increased to 30 patients to detect a 16% increase in GFR, in the present study, at a power of 0.8. The fact that filtration fraction was not altered with mannitol, however, suggests that GFR increased in proportion to the increase in renal plasma flow in the present study. If mannitol affected only RBF, one would have expected a decrease in the filtration fraction, which was seen in similar group of patients receiving low-dose dopamine, which was found to increase RBF with no effects on the GFR [44]. Thus, we suggest that mannitol treatment in early AKI results in both vascular endothelial and tubular epithelial deswelling, which will improve both renal perfusion and filtration

Treatment of patients with AKI with mannitol did not affect the renal oxygen supply/demand relation, as assessed by no changes in renal oxygen extraction. Thus, the mannitol-induced increase in RBF was matched by a proportional increase in RVO_2_. It is well known that tubular sodium reabsorption is a major determinant of RVO_2 _in humans [45], and it was shown previously that a close association exists between the GFR, tubular sodium reabsorption, and RVO_2 _in humans [22,27,46], and any agent that increases the GFR has the potential to increase the RVO_2 _[22,27,46]. If mannitol affected only RBF in the present study, with no increase in GFR or RVO_2_, one would have expected a decrease in renal oxygen extraction, as was seen with low-dose dopamine, which increased RBF with no effects on the GFR or the RVO_2 _[44].

This study has several limitations. One major limitation is that we did not include a time-control group. One could, therefore, argue that changes in the measured renal or hemodynamic variables were not entirely caused by mannitol itself, but also, to some extent, by spontaneous fluctuations or time-dependent effects on these variables. Conversely, data on renal and systemic hemodynamics, as well as on renal function and oxygen metabolism, obtained during the two control periods, did not differ significantly. We, therefore, believe that the effects of mannitol on the measured renal variables in the present study are caused by mannitol and not by spontaneous fluctuations or time-dependent changes of these variables. Another limitation of this study is the relatively small sample size, as discussed earlier. A much larger population of patients must be studied to evaluate whether mannitol may improve renal outcome in AKI.

The obvious advantages with the continuous renal vein thermodilution technique are that repeated and rapid estimations of RBF can be performed at the bedside at short intervals. The thermodilution technique is validated against the gold-standard technique, which is the urinary clearance of PAH, corrected for by renal extraction-fraction of PAH [23]. It is neither dependent on a steady state, nor affected by extrarenal elimination or by changes in renal extraction. The thermodilution technique can, hence, be used in intensive care patients to detect dynamic changes in RBF.

## Conclusions

In the present study of patients with postoperative AKI caused by severe heart failure, requiring inotropic and mechanical support, we showed that treatment with the osmotic diuretic, mannitol, induces a renal vasodilation and increases RBF with maintained filtration fraction and renal oxygenation.

## Key messages

Mannitol in the treatment of postoperative ischemic AKI

• causes renal vasodilation with a 12% increase in renal blood flow

• redistributes systemic blood flow to the kidneys

• maintains renal filtration fraction (that is, causes a balanced increase in GFR and renal plasma flow)

• maintains the renal oxygen supply/demand relation (that is, the increase in renal blood flow was matched by a proportional increase in renal oxygen consumption)

## Abbreviations

ACE: angiotensin-converting enzyme; BSA: body surface area; CABG: coronary artery bypass surgery; CI: cardiac index; CPB: cardiopulmonary bypass; CVP: central venous pressure; FENa: fractional excretion of sodium; FF: filtration fraction; GFNa: sodium filtration; GFR: glomerular filtration rate; Hct: hematocrit; HR: heart rate; IABP: intraaortic balloon pump; ICU: intensive care unit; LVEF: left ventricular ejection fraction; MAP: mean arterial pressure; MPAP: mean pulmonary artery pressure; PCWP: pulmonary capillary wedge pressure; preop: preoperative; PVRI: pulmonary vascular resistance index; RBF: renal blood flow; RO_2_Ex: renal oxygen extraction; RVO_2_: renal vascular oxygen consumption; RVR: renal vascular resistance; SOFA: sequential organ-failure assessment; SVI: stroke volume index; SVRI: systemic vascular resistance index; TRNa: tubular sodium reabsorption.

## Competing interests

The authors declare that they have no competing interests.

## Authors' contributions

All authors participated in the study design. GB collected and prepared the data and performed the statistical analysis. GB and BR performed the renal vein catheterizations and the experimental procedures. All authors participated in writing the paper, and all approved the final manuscript.
